The article "Predictive Value of CT Perfusion Imaging on the Basis of Automatic Segmentation Algorithm to Evaluate the Collateral Blood Flow Status on the Outcome of Reperfusion Therapy for Ischemic Stroke" was retracted in 2023. Reasons: signs of a paper mill; compromised peer review; unreliable results or conclusions.

# Predictive Value of CT Perfusion Imaging on the Basis of Automatic Segmentation Algorithm to Evaluate the Collateral Blood Flow Status on the Outcome of Reperfusion Therapy for Ischemic Stroke

**DOI:** 10.1155/2021/4463975

**Published:** 2021-11-11

**Authors:** Qingsong Gong, Botao Yu, Mengjie Wang, Min Chen, Haowen Xu, Jianbo Gao

**Affiliations:** ^1^Department of Radiology, The First Affiliated Hospital of Zhengzhou University, Zhengzhou, Henan 450000, China; ^2^Department of Neurology, The First Affiliated Hospital of Zhengzhou University, Zhengzhou, Henan 450000, China; ^3^Department of Neurointervention, The First Affiliated Hospital of Zhengzhou University, Zhengzhou, Henan 450000, China

## Abstract

Our objective was to study the predictive value of CT perfusion imaging based on automatic segmentation algorithm for evaluating collateral blood flow status in the outcome of reperfusion therapy for ischemic stroke. All data of 30 patients with ischemic stroke reperfusion in our hospital were collected and examined by CT perfusion imaging. Convolutional neural network (CNN) algorithm was used to segment perfusion imaging map and evaluate the results. The patients were grouped by regional leptomeningeal collateral score (rLMCs). Binary logistic regression was used to analyze the independent influencing factors of collateral blood flow on brain CT perfusion. The modified Scandinavian Stroke Scale was used to evaluate the prognosis of patients, and the effects of different collateral flow conditions on prognosis were obtained. The accuracy of CNN segmentation image is 62.61%, the sensitivity is 87.42%, the similarity coefficient is 93.76%, and the segmentation result quality is higher. Blood glucose (95% CI = 0.943, *P*=0.028) and ischemic stroke history (95% CI = 0.855, *P*=0.003) were independent factors affecting the collateral blood flow status of stroke patients. CBF (95% CI = 0.818, *P*=0.008) and CBV (95% CI = 0.796, *P*=0.016) were independent influencing factors of CT perfusion parameters. After 3 weeks of onset, the prognostic function defect score of the good collateral flow group (11.11%) was lower than that of the poor group (41.67%) (*P* < 0.05). The automatic segmentation algorithm has more accurate segmentation ability for stroke CT perfusion imaging and plays a good auxiliary role in the diagnosis of clinical stroke reperfusion therapy. The collateral blood flow state based on CT perfusion imaging is helpful to predict the treatment outcome of patients with ischemic stroke and further predict the prognosis of patients.

## 1. Introduction

According to the statistics of the 2019 edition of the *Global Burden of Disease Study*, since the 1990s, stroke became the second disease resulting in death in the world, second only to heart disease, and the second leading cause of disability due to disease in the world [1–3]. More than 81 million persons worldwide suffer from stroke [4]. At present, the clinical diagnosis of patients with ischemic stroke mostly excludes the congenital brain injury caused by external factors and uses digital subtraction angiography to check the cerebral vascular system of patients. The feature of digital subtraction angiography (DSA) is that it can eliminate the redundant tissue structure and accurately retain the angiography after special treatment. Therefore, the information such as vascular status and blood flow direction can be observed. However, digital subtraction angiography requires radioactive substances and arterial intubation, which poses a greater risk to patients. Therefore, a method that will not cause trauma to patients, CT perfusion imaging technology, is widely used in clinical treatment. In clinical treatment, doctors will choose CT and MRI to distinguish and divide the focus of stroke. However, the artificially depicted lesion site will not only have subjective differences, resulting in inaccurate images, but also add additional workload to doctors. With the rapid development of artificial intelligence algorithm and the continuous updating of medical equipment, it is particularly important to apply the algorithm in the accurate division of lesion parts in the stroke image to help clinicians provide more suitable personalized treatment plan for stroke patients. The automatic segmentation algorithm of convolutional neural networks (CNNs) belongs to a multilevel supervised learning network structure algorithm. In this network structure, pooling layer and convolution layer are the two main parts, which work together to segment the target features in CNN [5, 6]. Some studies used the multichannel CNN model to accurately divide the brain tumors of patients from the brain MRI images. Moreover, these regions are also divided into brain necrosis regions, brain edema regions, and brain enhancement and nonenhancement regions. Finally, certain evaluation indicators are used, and it is found that MRI based on CNN algorithm can effectively divide the characteristic regions of brain tumors [7]. However, few data have applied CNN algorithm to the classification of lesions in stroke patients. Therefore, in this study, CNN algorithm was used to extract and segment the lesions from CT perfusion images of stroke patients.

If the brain structure feels that the oxygen supply in the blood flow is interrupted for more than 6 seconds, the activity of brain nerve cells will be abnormal. Within the next 15 seconds, the patient will show clinical symptoms of unconsciousness and blurred consciousness. Within 120 seconds, the patient's EEG will show that the amplitude of brain waves will decrease and the normal electrical activity of the brain will stop. If patients do not receive timely assistance within 300 seconds, irreversible normal brain function damage will occur, resulting in serious diseases such as cerebral infarction, cerebral thrombosis, and atherosclerosis. If the blocked or narrowed blood vessels in patients with ischemic stroke are reperfused in time to ensure that the blood vessels of the patients are quickly and effectively dredged, the brain infarction of the patients can be reduced [8, 9]. In clinical practice, intravenous thrombolysis is often used to treat ischemic stroke with vasodilator therapy [10]. However, for some patients who cannot receive thrombolytic therapy in time in the treatment window for various reasons or have contraindications to thrombolytic surgery, even after thrombolysis, the blood flow in the blood vessel cannot guarantee the reoccurrence of embolism. However, the blood flow of cerebral collateral circulation can supply blood to the blood vessels in the ischemic stroke area and restore the normal blood flow in the ischemic area [11–13]. Therefore, the blood flow status of cerebral collateral circulation is also of great significance in aspect of the ischemic stroke patients' treatment. However, there are few reports on the predictive value of collateral blood flow status in stroke patients and its impact on prognosis.

Based on this, this study intends to use an automatic segmentation algorithm based on convolutional neural networks to segment the CT perfusion image of ischemic stroke and compare different collateral blood flow conditions for reperfusion treatment of ischemic stroke. The predictive value of the outcome of the clinical CT perfusion imaging is expected to provide a reference for the prediction of the outcome of ischemic stroke reperfusion therapy in the evaluation of collateral blood flow status.

## 2. Methods

### 2.1. Research Objects

In this study, a total of 30 patients with ischemic stroke in the inpatient ward of neurology rehabilitation department of our hospital were selected as the research objects. There were 19 male patients and 11 female patients. The age ranged from 33 to 78 years, with a mean age of 55.5 years.

Inclusion criteria were as follows: (1) The patient's age ranged from 33 to 78 years. (2) The patient's condition was clearly diagnosed as ischemic stroke according to the 2019 *China Guidelines for the Diagnosis and Treatment of Acute Ischemic Stroke*. (3) All clinical data and information are complete, and it is the first onset without previous stroke history. (4) The patient has reperfusion indications and is receiving reperfusion therapy. (5) The patient had no other neurological lesions, such as intracerebral hemorrhage.

Exclusion criteria were as follows: (1) The patient's age is inconsistent. (2) The patient had other serious complications. (3) The patient had coagulation dysfunction. (4) The patient was allergic to contrast media and disinfectant alcohol. (5) The patient had mental problems or consciousness disorders and poor compliance.

In this study, informed consent was signed by all patients and their families, and the study was approved by the medical ethics committee of our hospital.

### 2.2. CT Perfusion Method

The scanning equipment is Siemens Definition 64-row CT scanner. The patient should lie flat and do not swallow or do other actions as much as possible, the head was fixed, no rotating, and the patient was informed with the possible discomfort symptoms in advance. When the inspection started, the scanning layer thickness and layer spacing were set to 6 mm, and the scanning current was set to 420 mA and the voltage to 120 KV for continuous scanning. Iohexol (manufacturer: GE Pharmaceutical Co., Ltd.) was selected as the contrast medium, with a dose of 50 mL and a rate of 5 mL/s. After 6 s, the basal ganglia were used as the central layer to start perfusion imaging scanning for 50 s.

### 2.3. Segmentation of CT Perfusion Imaging Images Based on CNN

For early auxiliary diagnosis and thrombolytic treatment of stroke patients, it is of great significance for clinicians to make early diagnosis and treatment for patients by accurately extracting and segmenting the patient's imaging lesions. The CNN image automatic segmentation algorithm is a method similar to the traditional neural network algorithm model that can be reversed and can effectively segment medical images. It mainly has several important modules: input layer, convolution layer, pooling layer, connection layer, and output layer. These levels are composed of different numbers of two-dimensional plane network models. Compared with the traditional neural network structure, the input data of CNN is usually in the form of image, and the network structure can be changed according to the input image data with certain spatial characteristics, so as to maximize the utilization of the input image data, reduce the setting of other auxiliary parameters, and speed up the processing time of neural network. The flow grid diagram of CNN image segmentation algorithm is illustrated in Figure 1.

As a network structure algorithm for automatic image segmentation and recognition, CNN can automatically divide the corresponding feature areas without extracting the target features in advance. The input layer is generally image mode, and the convolution layer's function is to extract image features. The mathematical calculation is shown in the following equation:

(1) $$\begin{array}{c} n_{j}^{X}=f\left(\sum_{i\in M}n_{j}^{X-1}*a_{ij}^{X}+m_{j}^{X}\right), \end{array}$$

where *n*_*j*_^*X*^ represents the output result. *f* represents the activation function. *n*_*j*_^*X*−1^ represents the output result diagram of X−1 layer (the previous layer). *∗* represents the specific convolution operation in the algorithm. *a*_*ij*_^*X*^ represents the weight of each convolution kernel, that is, the relative importance of the two-dimensional filter matrix on each convolution layer in the algorithm. *m*_*j*_^*X*^ represents offset; that is, the segmentation line does not pass through the origin, so that the segmentation range is larger. The process of CNN is to continuously adjust the weight and bias of the convolution kernel to make its output reach the expected value. The activation function is to map the extracted features to a specific space through the nonlinear function, that is, to improve the nonlinear effect. Activation functions generally include Sigmoid function and ReLu function. Mathematical equation of Sigmoid function and the mathematical equation of ReLu activation function are as follows:

(2) $$\begin{array}{c} \sigma \left(x\right)=\frac{1}{1+e^{-x}},\\ R\left(x\right)=\max\left(o,x\right)=\left\{\begin{array}{cc} x, & x\geq 0,\\ 0， & x<0. \end{array}\right. \end{array}$$

The function of pooling layer is to reduce the amount of parameter calculation in the network image, reduce the complexity, and improve the fault tolerance of the algorithm. The mathematical calculation method is as follows:

(3) $$\begin{array}{c} n_{j}^{X}=f\left(\alpha_{j}^{X}\text{sub }n_{j}^{X-1}+\beta_{j}^{X}\right), \end{array}$$

where *α*_*j*_^*X*^ represents a multiplicative bias, sub represents the downsampling function, that is, the image is specifically reduced by function, and *β*_*j*_^*X*^ represents additive bias.

The pooling operation of pooling layer is divided into three types: average pooling, maximum pooling, and random pooling. The maximum pooling operation is usually used to output the pooling layer (Figure 2).

### 2.4. Evaluation Index for Segmentation Results of CT Perfusion Imaging

In order to evaluate whether CNN automatic segmentation algorithm can accurately segment the images of CT perfusion ischemic stroke patients, three indexes of precision (PRE), sensitivity (SEN), and Dice similarity coefficient (DSC) were used for quantitative evaluation. The accuracy represented the ratio of the correct segmentation area to the total segmentation area. Sensitivity represented the ability of image segmentation target feature region. ASD was the fineness of image segmentation. The larger the PRE, SEN, and DSC, the more accurate and the more valuable the segmentation result of the image. The calculation method is as follows:

(4) $$\begin{array}{c} \text{PRE}=\frac{TP}{TP+FP},\\ \text{SEN}=\frac{TP}{TP+FN},\\ \text{DSC}=\frac{2\left|M\cap^{}N\right|}{\left|M\right|+\left|N\right|}, \end{array}$$

where TP represents true positive (the segmentation results are true lesions and actually true lesions), FP indicates false positive (the segmentation results are true lesions, but not actually lesions), FN represents false negative (the segmentation results are not lesions but actually lesions), *M* represents the segmentation result of the lesion by the radiologist, and *N* is the lesion segmentation result of automatic segmentation algorithm.

### 2.5. rLMCs Collateral Blood Flow Status Scoring Method

rLMCs scoring standard is as follows: 0: no blood flow signal and noise; 1 point: there are few collateral blood flow signals in diastole; 2 points: the diastolic collateral blood flow is basically the same as that of the other side; 3 points: there is blood flow signal and the average flow velocity is enhanced; 4 points: the number of vascular development increases; 5 points: the blood flow and blood flow velocity are normal. Among them, 0–1 points is set as complete vascular occlusion. 2–3 points are set as the partial recanalization of blood vessels. From 4 to 5 points, the blood vessels are completely unobstructed. The total score ≤3 means poor collateral blood flow, and the total score >4 means good collateral blood flow.

All scoring results of this time shall be carried out independently by two imaging doctors. In case of great differences of opinion, it shall be submitted to the third imaging doctor for evaluation and finally reach an agreement.

### 2.6. CT Perfusion Parameters and Prognostic Evaluation Indicators

The CT perfusion parameters of the two groups were compared, including cerebral blood flow (CBF), cerebral blood volume (CBV), mean transit time (MTT), and time to peak (TTP) to observe collateral blood flow and the influence of the condition on ischemic stroke. In addition, the modified Scandinavian Stroke Scale was used as a prognostic index to evaluate the effect of collateral blood status on the outcome of reperfusion therapy in patients with ischemic stroke.

### 2.7. Statistical Analysis

SPSS 20.0 statistical software was used to analyze data of this study. The measurement data in line with normal distribution were analyzed by one-way variance method, x^2^ test was used to analyze the counting data, and the selected univariate factors used logistic regression analysis to determine the factors of collateral circulation status on the outcome of stroke reperfusion treatment. *P* < 0.05 represented the fact that the difference was statistically significant.

## 3. Results

### 3.1. Segmentation Results of CT Perfusion Imaging Based on CNN

The CNN automatic segmentation algorithm is used to segment the CT perfusion image of ischemic stroke. The results of this segmentation algorithm are compared with the region growth algorithm [14].  Figure 3(a) shows the original imaging of a patient with ischemic stroke.  Figure 3(b) shows the results of segmentation using the algorithm in this study.  Figure 3(c) indicates the segmentation results of the region growth algorithm method. The image in Figure 3(b) is clearer and has higher resolution, clearer boundary, and better segmentation quality relative to Figure 3(c).

### 3.2. Segmentation Result Evaluation Index

To quantitatively evaluate the segmentation results, PRE, SEN, and DSC are used in evaluation. The algorithm of this study is compared with the region growth algorithm. The results show the algorithms PRN, SEN, and DSC used in this study are 62.61%, 87.42%, and 93.76%. Relative to the region growing algorithm, the three indexes of CNN automatic segmentation algorithm are improved, the accuracy and similarity coefficient are doubled, and the sensitivity is increased by 1.1 times. As can be concluded from Table 1, the algorithm adopted in this study has a better segmentation effect on CT perfusion images.

### 3.3. Collateral Blood Flow Score and Basic Data of All Patients

There were 30 patients in this study. According to the rLMCs score index, the collateral blood flow status of 30 patients was grouped. There were 18 patients with rLMCs total score >4, and 12 patients with rLMCs total score ≤3. Therefore, 18 patients with total score >4 were set as the good collateral blood flow status group, and 12 patients with total score ≤3 were set as the poor collateral blood flow status group. Compared with the good group, there were significant differences in blood glucose, ischemic stroke history, and family history in the bad group (*P* < 0.05) (Table 2).

### 3.4. Independent Influencing Factors of Collateral Blood Flow Status

Logistic regression analysis was used to analyze the three influencing factors of blood glucose, history of ischemic stroke, and family history in the table. The results showed that blood glucose and history of ischemic stroke were independent factors affecting collateral blood flow status of stroke patients (Table 3).

### 3.5. Factors Influencing CT Perfusion Parameters

After CT perfusion imaging, four indexes were used to evaluate the results in the good group and the bad group. CBF, CBV, and MTT in the group with good collateral circulation were obviously higher relative to poor collateral circulation group, and there was significant difference between CBF and CBV (*P* < 0.05). Moreover, the TTP of the good group was also lower in the two groups. It is suggested that the cerebral ischemia status of patients with ischemic stroke can be reflected by evaluating the blood status of cerebral collateral branches, which has predictive value for the outcome of ischemic stroke reperfusion treatment (Figure 4).  Figure 4(a) represents the comparison of CBF values.  Figure 4(b) is the comparison of CBV values.  Figure 4(c) shows the comparison of MTT values.  Figure 4(d) represents the comparison of TTP values.

By incorporating CBF and CBV into binary logistic regression analysis, it was found that the AUC of CBF was 0.865, and that of CBV was 0.822. The two factors had significant effects on CT perfusion parameters, thus further quantitatively reflecting the outcome of reperfusion therapy for ischemic stroke. It is suggested that CBF and CBV of collateral vessels are correlated with the prognosis of patients with ischemic stroke after reperfusion (Table 4).

### 3.6. Comparison of Prognosis Function Defect

Scoring after Scandinavian Stroke Scale was modified. It was stipulated that patients with clear consciousness, basically normal communication, basically complete normal eye rotation, and mild or no facial paralysis symptoms were normal. Patients with unclear consciousness, who are unable to speak, unable to see the specified field of vision, and with unilateral or bilateral facial paralysis were set as severe. The results showed that, three weeks after onset, the scores of patients with poor cerebral collateral blood circulation were significantly lower than those with good collateral blood circulation (*P* < 0.05). The results were as follows (Table 5).

## 4. Discussion

Stroke is divided into ischemic stroke and hemorrhagic stroke. Ischemic stroke is a kind of brain disease with high mortality and disability rate in cardiovascular and cerebrovascular diseases, accounting for about 70% of the incidence of cardiovascular and cerebrovascular diseases. About 84.4% of the more than 81 million global stroke patients had ischemic stroke [15]. For the early diagnosis and treatment of stroke, in order to better identify the location of the lesion, imaging doctors need to divide the image processing. At present, the segmentation of lesions in the image of patients with ischemic stroke is usually manually segmented by professional imaging doctors. The segmentation results depend on the doctor's medical knowledge and clinical experience and have strong subjectivity. Different imaging doctors segment lesions differently. Artificial segmentation of the lesion is time-consuming and laborious, and as more medical images need to be processed, an imaging doctor obviously cannot meet the needs of lesion segmentation. With the continuous improvement of computer technology and medical equipment, an automatic segmentation algorithm based on CNN becomes a research hotspot. This algorithm can not only quickly assist doctors to identify the lesion site of stroke but also automatically divide the lesion site, which is convenient for doctors to locate the lesion area directly through imaging observation and provides great help for subsequent treatment [16]. In this study, CNN automatic segmentation algorithm and region growth algorithm are used to segment the CT perfusion image of stroke patients. The results revealed that, compared with the segmentation results of region growth algorithm, the segmentation results of this algorithm had clearer image, higher resolution, clearer boundary, and better segmentation quality. The image accuracy and similarity coefficient were doubled, and the sensitivity was increased by 1.1 times. This shows that CNN algorithm has a relatively accurate segmentation ability, which plays a good auxiliary role in the diagnosis of clinical stroke reperfusion therapy.

Collateral blood circulation in the brain mainly refers to that when the arteries and vessels in the brain are narrow or completely blocked, the rest of the normal collateral circulation in the brain can be used to help complete the blood supply, prevent the occurrence of ischemic penumbra, reduce the possibility of cerebral infarction, and avoid ischemic stroke. Therefore, collateral blood flow status is extremely important for the treatment of ischemic stroke. In the early reperfusion treatment of stroke, cerebral collateral circulation can not only improve the success rate of intravenous thrombolysis but also help patients with endovascular treatment in successful reperfusion. It has attracted more and more attention in helping patients reduce the risk of bleeding transformation and effectively improve the prognosis of patients. Studies showed that, in stroke patients with good cerebral collateral blood flow status, the blood perfusion TICI grade after reperfusion is relatively high, which is mainly related to the good prognosis of patients. In stroke patients with poor collateral blood flow status, the blood perfusion TICI grade cannot benefit the prognosis of patients [11]. However, there are great differences in collateral blood flow among patients with ischemic stroke. Nannoni et al. [17] found that age, dyslipidemia, and creatinine levels had a greater impact on collateral blood flow through general data analysis of patients with ischemic stroke. This study also found that blood glucose (95% CI = 0.943, *P*=0.028) and history of ischemic stroke (95% CI = 0.855, *P*=0.003) were independent factors affecting the collateral blood flow status of stroke patients.

There are many factors affecting the severity of ischemic stroke patients. In addition to the influence of collateral blood flow, the perfusion in the brain of patients is also important. Cerebral CT perfusion imaging can most intuitively reflect the blood flow status of the patient's brain, which can be used as an indicator of whether the brain tissue is ischemic [18]. The perfusion parameters of cerebral perfusion imaging in patients with ischemic stroke have additional important value for the outcome of clinical treatment. On the one hand, the quantitative analysis is performed to cerebral perfusion parameters; on the other hand, the perfusion pseudocolor map can also be qualitatively analyzed. These two aspects are combined to comprehensively evaluate the cerebral ischemic area, ischemic degree, and perfusion status of blood flow in patients with ischemic stroke, so as to provide the most reliable basis for clinical treatment. CBF can be used as an indicator to reflect the reserve capacity of cerebral blood flow circulation, CBV can be used as an indicator to indicate the cerebrovascular volume, and MTT can be used as an indicator to reflect the CT perfusion pressure of brain tissue. When MTT is prolonged, it means that the CT perfusion pressure of brain is reduced. As the time parameter of brain tissue, the prolongation of TTP indicates the time when the contrast agent is injected to the highest concentration and the outflow time is prolonged, indicating that the blood flow velocity of brain tissue is slowed down [19]. Therefore, cerebral CT perfusion imaging parameters are of great significance for patients with ischemic stroke receiving reperfusion therapy. The collateral blood flow of stroke patients is closely related to cerebral perfusion. Studies showed that rCBF, rCBV, and Tmax can independently predict collateral blood flow and are negatively correlated with the volume of stroke infarction [20]. The results of this study are consistent with the report. CBF (95% CI = 0.818, *P*=0.008) and CBV (95% CI = 0.796, *P*=0.016) were independent influencing factors of CT perfusion parameters. When the blood vessels in the patients with poor collateral blood flow conditions were narrowed, the blood flow in the brain tissue had changed significantly. The blood flow decreased within a certain period of time, and the blood flow velocity also gradually slowed down. The CT attention parameters were reflected in the decrease of CBF and the prolongation of MTT and TTP. It is suggested that CBF and CBV are better in patients with good collateral circulation, cerebral infarction is small, and good collateral blood flow can be used for bypass perfusion in ischemic penumbra.

Reports showed that, in patients with ischemic stroke before reperfusion therapy, the better the collateral blood flow, the smaller the risk of adverse reactions in patients with prognosis. Therefore, for patients with stroke who cannot be examined by MRI imaging, reperfusion therapy can be assisted by collateral blood flow status of patients [21]. In this study, it was found that, after 3 weeks of onset, the prognostic function defect score of the good collateral flow group was 11.11%, which was lower than that of the poor collateral flow group (41.67%), and the difference was significant (*P* < 0.05). This is basically consistent with the above reports.

## 5. Conclusion

As a kind of automatic segmentation algorithm, the accuracy, sensitivity, and similarity coefficient of CNN algorithm for lesion segmentation of patient perfusion imaging are 62.61%, 87.42%, and 93.76%, respectively. Compared with the results of the region growing algorithm, the results of the three indicators of image quality have at least doubled, and the image resolution has also increased, indicating that the CNN algorithm has more accurate segmentation ability for stroke CT perfusion imaging and plays a good auxiliary role in the diagnosis of clinical stroke reperfusion therapy. In addition, this study found that blood glucose (95% CI = 0.943, *P*=0.028) and ischemic stroke history (95% CI = 0.855, *P*=0.003) were independent factors affecting the collateral blood flow status of stroke patients by binary regression analysis. CBF (95% CI = 0.818, *P*=0.008) and CBV (95% CI = 0.796, *P*=0.016) were independent influencing factors of CT perfusion parameters. After 3 weeks of onset, the prognostic function defect score of patients with good collateral blood flow was 11.11%, which was lower than that of the poor group (41.67%), and the difference was significant (*P* < 0.05). It is suggested that collateral blood flow status has predictive value for stroke treatment process from the basic data of patients (blood glucose, history of ischemic stroke) and CT perfusion and further predicts the treatment outcome of patients.

## Figures and Tables

**Figure 1:** Basic structure of CNN automatic segmentation algorithm.

**Figure 2:** Maximum pool operation diagram.

**Figure 3:** Segmentation results of different algorithms.

**Figure 4:** Pathological evaluation indexes. (a) The comparison of CBF values between good group and bad group. (b) The comparison of CBV values between the groups. (c) The comparison of MTT values between two groups. (d) The comparison of TTP values between groups. *∗*When *P* < 0.05, the difference is statistically significant.

**Table 1:** Segmentation result evaluation index.

Algorithm type	PRE (%)	SEN (%)	DSC (%)
Automatic segmentation algorithm	60.61	98.42	93.76
Region growing algorithm	59.37	87.14	90.50

**Table 2:** Basic information of the patient.

Category	Good group (*n* = 18)	Bad group (*n* = 12)	*P*
Male	15	4	0.370
Age	53.11 ± 7.32	58.06 ± 4.83	0.553
Blood sugar	18	7	0.027
Smoking	8	9	0.175
Hypertension	16	13	0.742
Medical history	9	12	0.003
Family history	18	13	0.011
Diabetes (*n*)	7	5	0.084

**Table 3:** Binary logistic factor analysis results of influencing factors of collateral blood flow status.

Category	AUC	95% CI	*P*
Abnormal blood sugar	0.827	0.943	0.028
History of stroke	0.831	0.855	0.003
Family history	0.820	0.702	0.664

**Table 4:** Binary logistic influencing factors of CT perfusion parameters.

Category	AUC	95% CI	*P* value
CBF	0.865	0.818	0.008
CBV	0.822	0.796	0.016

**Table 5:** Statistical results of two groups of patients' score.

Group	Admission check		3 weeks after onset	
	Mild to moderate	Severe	Mild to moderate	Severe
Good group (*n* = 18)	11 (61.1%)	7 (38.9%)	16 (88.9%)	2 (11.1%)
Bad group (*n* = 12)	10 (83.3%)	2 (16.7%)	7 (58.3%)	5 (41.7%)
*P* value	0.078	0.236	0.003	0.045

## Data Availability

The data underlying the results presented in the study are included within the manuscript.
